# TCMNER and PubMed: A Novel Chinese Character-Level-Based Model and a Dataset for TCM Named Entity Recognition

**DOI:** 10.1155/2021/3544281

**Published:** 2021-08-07

**Authors:** Zhi Liu, Changyong Luo, Zeyu Zheng, Yan Li, Dianzheng Fu, Xinzhu Yu, Jiawei Zhao

**Affiliations:** ^1^University of Chinese Academy of Sciences, Beijing 100049, China; ^2^Shenyang Institute of Automation, Chinese Academy of Sciences, Shenyang 110016, China; ^3^Institutes for Robotics and Intelligent Manufacturing, Chinese Academy of Sciences, Shenyang 110016, China; ^4^Department of Infectious Diseases, Dongfang Hospital of Beijing University of Chinese Medicine, Beijing 100078, China; ^5^Education Section, Dongzhimen Hospital of Beijing University of Chinese Medicine, Beijing 101121, China; ^6^School of Information Science and Engineering, Shenyang University of Technology, Shenyang, China; ^7^College of Electrical Engineering, Zhejiang University, Hangzhou 310027, China

## Abstract

Intelligent traditional Chinese medicine (TCM) has become a popular research field by means of prospering of deep learning technology. Important achievements have been made in such representative tasks as automatic diagnosis of TCM syndromes and diseases and generation of TCM herbal prescriptions. However, one unavoidable issue that still hinders its progress is the lack of labeled samples, i.e., the TCM medical records. As an efficient tool, the named entity recognition (NER) models trained on various TCM resources can effectively alleviate this problem and continuously increase the labeled TCM samples. In this work, on the basis of in-depth analysis, we argue that the performance of the TCM named entity recognition model can be better by using the character-level representation and tagging and propose a novel word-character integrated self-attention module. With the help of TCM doctors and experts, we define 5 classes of TCM named entities and construct a comprehensive NER dataset containing the standard content of the publications and the clinical medical records. The experimental results on this dataset demonstrate the effectiveness of the proposed module.

## 1. Introduction

In recent years, with the booming of deep learning models, the applications of artificial intelligence technology in traditional medicine have achieved numerous achievements [1–3]. As a representative of traditional medicine, intelligent traditional Chinese medicine (TCM) has become a focused area. Many excellent works have been made in intelligent TCM such as TCM syndrome diagnosis based on symptom sequence [4–7], TCM herbal prescription generation [8, 9], and TCM disease diagnosis [10–12]. Currently, the models for realizing these intelligent TCM tasks mainly rely on the labeled samples. One of the biggest issues that urgently need to be solved is the lack of publicly available labeled samples, i.e., the TCM medical records. The TCM medical records contain the necessary items for realizing the TCM tasks mentioned above, including the clinical manifestation of a patient, the syndrome and disease diagnosis and treatment laws provided by the TCM doctor, and the herbal prescription prescribed by TCM doctor. How to automatically identify and extract these mentioned items from the TCM medical records by deep learning models is an efficient way to continuously increase labeled TCM samples. The named entity recognition (NER) model which aims to identify the target entity from the text is a useful method to solve the above issue. Several TCM NER studies are proposed in recent years with various purposes [13–21]. However, an unavoidable fact is that the previous works only focus on a specific TCM resource. The target resources are either in the standard publications [16, 17] or the clinical electronic medical records [13, 15, 19–21]. Different types of TCM resources pose different challenges for researchers. In general, it is much less difficult to identify the named entities that appear in TCM publications than in clinical electronic medical records. To our best knowledge, no study has been proposed to deal with the TCM NER task on publications and the clinical electronic medical records simultaneously, mainly due to the lack of the dataset that contains both these two types of data. In addition, according to our observation, the previous works of TCM NER are mainly focused on partial aspects (usually 2-3) of TCM. The classification of the TCM NER types is also not proper.

To fill the gaps in the dataset and the classification of TCM named entity, in this work, we collaborate with the doctors and experts from Beijing University of Chinese Medicine to define 5 classes of named entities, i.e., clinical manifestation, disease, herb, syndrome, and treatment law. These classes include all types of terms that may appear in the process of TCM diagnosis and treatment. We also propose a Chinese character-level traditional Chinese medicine NER model, called TCMNER, and a NER dataset for TCM. The dataset is collected by ourselves and contains both the publications and clinical electronic medical records from various types of TCM resources (e.g., articles, electronic medical records, and books). The TCMNER makes use of the Chinese character-level representation, aiming to realize a comprehensive TCM NER task. The reason why we use the Chinese character-level representation is that TCM terms usually are of variable length, especially the clinical manifestation term, which poses great challenges for the TCM NER task. In the TCM terminology, especially the clinical, TCM doctors usually use a phrase or a short sentence to record a symptom of a patient for describing the symptom in as much detail as possible. This kind of TCM term usually contains more than 6 Chinese characters existing in a sentence. Since there is no separator between Chinese words, the commonly used method is to segment the sentence first and then extract the TCM terms. The sentence segmentation may divide the term that should be kept as a word into several parts, which will miss the necessary part of the term or label the wrong tags when the auto-tagging process is used, leading to the semantic fault. Besides, the performance of such Chinese NER models is largely dependent on the segmentation results. Therefore, in this work, we argue that the character-level representation should be used for the TCM NER task. To relive the issue of lacking word/phrase semantic in the character-level representation, we propose a word semantics and word-character semantic relation integrating character-level representation strategy. The contributions of this work are summarized as follows:

- We define and classify the TCM named entity into 5 classes according to the classification of TCM and the process of TCM diagnosis and treatment, called **CSDTH** classification, including **C**linical manifestation, **S**yndrome, **D**isease, **T**reatment Law, and **H**erb.
- We collect and construct a comprehensive NER dataset called PubMed, which consists of both standard contents of the publications and the clinical electronic medical records from various TCM resources.
- We propose a novel Chinese character-level representation strategy for the TCM NER task.
- We conduct a series of comprehensive experiments to verify the performance of the proposed models. The experimental results demonstrate that the proposed Chinese character-level representation can improve the models' performance with a prominent margin.

### 1.1. Related Works

For alleviating the lack of the labeled NER sample, Wang et al. replaced the words in the training set with synonyms. A pretrained model was obtained on the augmented training set. Then the prior semantic knowledge learned by the pretrained model was transferred to the downstream NER task [15]. Zhang et al. considered the distant supervision to substitute the human annotation and propose a novel back-labeling approach to deal with the potential challenge of entities that are not included in the vocabulary [14]. Qu et al. focused on the fuzzy entity recognition problem and proposed the Bert-BiLSTM-CRF model. Their proposed model has an advantage in identifying drug names [17]. Knowledge graph information is utilized by Jin et al. to tackle the rare-word recognition problem. They proposed the TCMKG-LSTM-CRF model which introduces a knowledge attention model to apply the attention mechanism between the hidden vector of neural networks and knowledge graph candidate vectors. This model also takes the influence of previous words in a sentence into consideration [21]. Song et al. paid attention to the lexicon information of the target sentence. They incorporated the lexicon information into the representation layer of the BiLSTM-CRF. Experiments conducted on the “Shanghan Lun” dataset showed the outperformance of their method [16]. As for NER from Chinese electronic medical records, Gong et al. implemented a deep learning pretraining method, including word embedding and fine-tuning, as well as the BiLSTM and Transformer. This method identified four types of clinical entities including diseases, symptoms, drugs, and operations [19]. Liu et al. combined the BiLSTM-CRF model with semisupervised learning to reduce the cost of manual annotation and leveraged extraction results. The proposed method is of practical utility in improving the extraction of five types of TCM clinical terms, including traditional Chinese medicine, symptoms, patterns, diseases, and formulas [22]. Zhang et al. worked on building a fine-grained entity annotation corpus of TCM clinical records [13]. They exploited a four-step approach: (1) determine the entity types through sample annotation, (2) draft a fine-grained annotation guideline, (3) update the guidelines until the prospective performance is achieved, and (4) use the guidelines developed in steps 2 and 3 to construct corpus. Yin et al. pointed out the drawbacks of the BiLSTMs model in NER such that this method can only capture contextual semantics between characters in sentences. Thus, they improved the BiLSTM-CRF model with the use of the radical-level feature and self-attention mechanism. Results of the experiments show comparable performance [20]. As we discussed, a commonly used underlying method in the previous studies is the segmentation of the target sentence. It leads to the wrong tokens and the words with incomplete semantics. Besides, a comprehensive NER dataset and named entity schema in TCM are still not presented. In this study, we focus our attention on addressing these issues.

## 2. Materials and Methods

### 2.1. Traditional Chinese Medicine Named Entity Definition

In this work, we collaborate with the doctors and experts from Beijing University of Chinese Medicine and Dongzhimen Hospital of Beijing University of Chinese Medicine to define and classify the TCM named entity systematically and comprehensively. After a throughout analysis of the previous works, we found that the classes of TCM named entity that are used in the previous works usually only consider partial types of TCM terms [15, 16]. Some works subdivide one class of TCM named entity into several subclasses [13]. We analyse the TCM basic theory, different branches of TCM, and the terms used in the process of TCM clinical diagnosis and treatment, summarizing the TCM named entities into 5 classes. The summarized classes contain **C**linical manifestation, **S**yndrome, **D**isease, **T**reatment law, and **H**erb, **CSDTH** for short.

As shown in Table 1, this is an example of the TCM-related clinical records. These 5 classes cover almost all aspects of TCM. For instance, the clinical manifestation entities contain all symptoms of a patient collected by the TCM doctor through four ways of diagnosis, namely looking (red tongue, less tongue coating), listening (wheezing due to retention of phlegm in throat), questioning (insomnia, dreaminess, palpitation, dry stool and once every 2 days, amnesia, tidal fever, and night sweating), and feeling the pulse and skin (small and weak pulse). It is worth noting that, in this work, the symptoms of tongue and pulse, e.g., red tongue and small and weak pulse, and systemic symptoms such as insomnia, dreaminess, and palpitation fall into the same category of clinical manifestation. According to the advice of the TCM doctors and experts, the symptoms of tongue and pulse belong to the symptom category, so that there is no need to subdivide them into subcategories. Another difference between this work and the previous works in the class of TCM named entity is the herb. In this work, we enable the model to identify the most valuable treatment unit—the herb instead of the prescription name, because, in the downstream TCM AI tasks such as the TCM prescription generation, the model needs to capture the interaction between symptoms and herbs and generate a set of or sequence of herbs to form a TCM herbal prescription. Therefore, the identification of herbs is much needed than the prescription name. Based on this named entity classification strategy, we explore the BIO schema to define the entity tags which are shown in Table 2.

### 2.2. Word-Character Integrated Self-Attention

As we discussed in introduction, we argue that the TCM NER should be accomplished by utilizing the Chinese character-level representation and tagging to maintain the complete semantics of the named entities of the long words, phrases, or short sentences. However, the character-level representation does not capture the word semantics and the phrase semantics. To alleviate this issue, we propose a novel module that can integrate the word-character semantic relation and word semantics into character-level representation, outputting the character-level representation with word semantics and word-character semantic relation. The overall architecture of the module is shown in Figure 1.

As shown in Figure 1, the character-level and word/phrase-level representations are obtained by the embedding layers. Then, an attention module takes the word representation and character-level representation as input to output the attention weights **e**_**j**_ to each character in the word/phrase. Each attention weight *e*_*j*_^*i*^ represents, according to the word/phrase semantic, the importance of *i*-th character in the given word/phrase. When the attention weights are gained, the module can generate the word semantic and word-character semantic relation integrating character-level representation. The operations of this process are formulated as follows:

(1) $$\begin{array}{c} R_{\text{word}}=\text{Embedding}\left(x_{\text{word}}\cdot W_{\text{word}}\right),\\ R_{\text{character}}=\text{Embedding}\left(x_{\text{character}}\cdot W_{\text{character}}\right),\\ e_{j}=\text{soft max}\left(R_{\text{word}}\cdot W_{\text{attn}}\cdot R_{\text{character}}+b_{\text{attn}}\right),\\ \text{soft max}=\frac{\exp\left(x_{t}\right)}{\sum_{j=1}^{T}\text{erp}\left(x_{j}\right)}, \end{array}$$

where *W*_*∗*_ and *b*_*∗*_ means the trainable parameters and *R*_character_ contains *l* vectors. After the attention weights are obtained, the new character level for each char is calculated as the weighted sum of *R*_character_, i.e., *R*_character_^*i*^=∑_*i*=1_^*l*^*e*_*j*_^*i*^ × [*R*_character_^*i*^, *R*_word_^*i*^].

Notice that the Embedding and attention operations are agnostic to the model; researchers can replace these two operations with any applicable functions, such that the Embedding operation can be replaced by the popular pretraining language models (e.g., BERT and ALBERT), so does the attention operations. In this work, the multihead self-attention operation is used to capture the word semantics, the word-pieces semantics, and the word-character semantic relations. How to apply the multihead self-attention to generate the new character-level representation based on the word- and character-level representation is shown in Figure 2. The self-attention module takes the character-level representation as its *key* and *value*, and the word/phrase-level representation as its *query*. In this way, the information of word/phrase and character can interact with each other, and the new character representation can be generated by fusing these two types of information. This module is a plug-and-play unit that is readily combined with the other models to do the TCM NER task. We will verify its effectiveness and efficiency in the next section in detail.

## 3. Results and Discussion

### 3.1. Datasets and Metrics

As we discussed before, due to the limited availability of TCM resources, there is no comprehensive TCM NER dataset that contains both standard publications and the clinical medical records. To fill this gap, with the help of doctors and experts from Beijing University of Chinese Medicine and Dongzhimen Hospital of Beijing University of Chinese Medicine, we first collect the standard content of the books including the *Basic Theory of Traditional Chinese Medicine*, the *Diagnostics of Traditional Chinese Medicine*, the *Surgery of Traditional Chinese Medicine*, the *Traditional Chinese Pharmacology*, and the open accessed TCM articles. We omit the unnecessary content of these publications and only retain the text. Then, all retained texts are split into sentences of which each sentence is regarded as a NER sample. The desensitized clinical medical records are provided by Dongzhimen Hospital of Beijing University of Chinese Medicine. We retain the terms of clinical manifestation, syndrome diagnosis, disease diagnosis, treatment law, and herbs (the herbs in the prescription, not the prescription name) from each medical record. We combine these two datasets as the entire dataset. The statistics of the dataset is shown in Tables 3 and 4. This comprehensive dataset contains 94380 samples in total. We split the dataset into training, validation, and test sets with the proportion of 6 : 2 : 2. The samples of clinical manifestation, syndrome, disease, treatment law, and herb in the training set are 24332, 7613, 2808, 11186, and 11682, respectively. The total samples of these 5 classes are larger than the 94380, because some of the samples both contain multiple types of entities.

We also calculate the number of the 5 classes for each dataset. As shown in Table 4, we notice that in both datasets the most common entity type is the clinical manifestation. In the publication dataset and medical record dataset, there are 18150 and 75177, respectively. Medical records contain more entities than publications. The reason is that there is a great deal of content in publications to explain and prove the theories and results. We also note that the number of disease entities is the lowest in both datasets. We count the samples for each dataset and notice that the although number of samples in the medical record dataset is less than the publication dataset, the number of entities of all classes in the medical record dataset is far more than the publication dataset. It demonstrates that the medical record contains more effective entities than the publications in each sample.

In this work, we conduct a series of comprehensive experiments to verify the proposed module. The comparison models include (1) BiLSTM-CRF, a bidirectional long-short term memory network (LSTM) with conditional random field (CRF) layer that is the most popular architecture for NER task before the appearance of pretrained language models; (2) BERT, a commonly used language model that can generate a bidirectional contextual representation for the NLP downstream tasks; (3) BERT-LSTM, a BERT model combined with the LSTM; (4) BERT-CRF, a BERT model combined with a CRF layer; (5) BERT-BiLSTM, a BERT model combined with a bidirectional LSTM; (6) BERT-BiLSTM-CRF, a BERT model combined with BiLSTM, and the CRF layer is followed; (7) RoBERTa, a BERT model with several adjustments, which achieves better performance on the downstream NLP tasks; (8) RoBERTa-LSTM, a RoBERTa model combined with a LSTM layer; and (9) RoBERTa-BiLSTM, a RoBERTa model combined with a bidirectional LSTM layer. All the comparison models are explored with different purposes. For evaluation metrics, we introduce the precision, recall, and F1-score. Precision refers to the ratio of correct entities to predicted entities. The recall is the proportion of the entities in the test set which are correctly predicted. The F1-score is a balanced measure of precision and recall and is calculated by the following formulation:

(2) $$\begin{array}{c} F1=\frac{2*\text{precision}*\text{recall}}{\text{precision}+\text{recall}}. \end{array}$$

The traditional way to calculate the values of precision, recall, and F1-score is based on the classification results of the NER model, which reflects the performance of the model in classifying samples into the desired category. In addition to the traditional classification evaluation, we introduce a rigorous method to calculate the values of precision, recall, and F1-score, called ***identification***. In TCM NER, in addition to the entities of the target class, there are plenty of entities marked with “O”. The entity labeled “O” is not a useful entity in real-world scenario. The models that can classify the target entities into their correct categories are much more important than the models correctly classifying the entities as “O”. Thus, in this kind of experiment, we filter out the “O” tags in each label and only retain the target 5-class entity tags and their positions in the original sample. The predicted tags are also filtered by these positions. In this way, we can focus our attention on verifying the models' performance to identify the useful types of entities. Since the aim of TCM NER is that the trained NER model can obtain a higher identification performance in new electronic medical records, we train all comparison models in publications first. Then, all models are evaluated in the medical records to verify their recognition performance. The publication dataset is also divided with the proportion of 6 : 2 : 2.

### 3.2. Experimental Results

We take the RoBERTa with word-character integrated self-attention model, called RoBERTa-c, as our basic model to compare with other models. We trained the BiLSTM-CRF, BERT-CRF, BERT-BiLSTM, BERT-BiLSTM-CRF, RoBERTa-BiLSTM, and RoBERTa-c to verify the performance of different models on the publication dataset. Then, the test set of publication and all samples in the medical record dataset are used for verification purposes. The precision, recall, and F1-score of all comparison models are shown in Table 5. As shown in Table 5, the BiLSTM-CRF model obtains a higher precision than BERT-CRF on both publications and medical records. This is inconsistent with researchers' intuition since the only difference between these two models is the representation extraction layer. The BERT's ability to extract the contextual representation is better than LSTM, which is proved in numerous studies, whereas the recall of BERT-CRF is far better than BiLSTM-CRF. Comparing the BERT-BiLSTM with BERT-BiLSTM-CRF, we notice that, without the CRF layer, the BERT-BiLSTM gains a significant improvement on both datasets. Combined with the performance of BERT-CRF and BiLSTM-CRF, the performance decrease of BERT-CRF and BiLSTM-CRF may be caused by the layer of CRF. The RoBERTa-BiLSTM obtains a similar result with BERT-BiLSTM on publication dataset but gains a better performance on medical record dataset, which gains a 1.4% F1-score. With the assistance of the proposed character representation, the best performance is obtained by using only RoBERTa among all comparison models. The F1-scores on both datasets are higher than 90%. It is noticed that, for all comparison models, almost all models obtain a higher precision, recall, and F1-score on the test set of publications than medical records except for the BILSTM-CRF.

To verify the generalization ability of the proposed word-character integrated self-attention module for all models compared in this work, we conduct the ablation studies of the whole models. We combine each model with the word-character integrated self-attention module and rename it as “*∗*-c,” where the “*∗*” represents the original model's name and “-c” means the word-character integrated self-attention module. In these experiments, we also verify each model's performance on every category of the TCM named entity. For each category, we only retain the samples that contain only one type of entities and filter out the samples that contain the other 4 types of entities, forming 5 distinctive datasets. The F1-scores for all models on 6 datasets are shown in Table 6.

As shown in Table 6, we notice that the performance of each model with the word-character integrated self-attention module is improved to a certain degree. Each model with the proposed module obtains a 1%-2% improvement on F1-score. We notice that the biggest improvement of performance is BERT-BiLSTM-CRF, which means that the word-character integrated self-attention module can effectively relieve the performance decrease caused by the CRF layer. Comparing BERT, BERT-LSTM, and BERT-BiLSTM, we found that the BERT obtains the best performance on all 6 datasets. Adding the LSTM layer following the BERT causes the performance decrease. The reason might be that the representation obtained by BERT already contains the bidirectional contextual information of the sentence/text. The LSTM layer can only use the semantic information in one direction, which erases the necessary information in the other direction. The reason we came to this assumption is that when the BiLSTM layer is used after the BERT, its performance is significantly improved. The same situation happened in the experiments of RoBERTa-based models. The RoBERTa obtains the best results on all 6 datasets when compared with RoBERTa-LSTM and RoBERTa-BiLSTM. The LSTM layer also causes the performance decrease on RoBERTa and the BiLSTM layer improves the performance back. Both models that only use the BERT and RoBERTa almost gain the highest F1-score among the other corresponding LSTM-based two architectures, which shows that the underlying language models can capture the good contextual representation from the target sentences. The BERT-c and RoBERTa-c demonstrate that the word-character integrated self-attention module can make it better. In this work, the experiments show that the LSMT layer, BiLSTM, and CRF layer may cause the performance decrease. For all datasets, we found that all models achieve poorer performances on the medical record dataset than the publication dataset. This may be caused by two reasons: (1) all models are trained on the training set of the publication dataset and fitted well on it and (2) the medical record datasets are the clinical electronic records whose terms are not filled and wrote very formally.

In real-world scenarios, the aim of TCM NER is to identify the useful named entities from the clinical electronic records, e.g., clinical manifestation, syndrome, disease, treatment law, and herb, instead of the unnecessary entities such as the patient's name and the patient's age. In the schema of NER, these unnecessary entities are tagged as “O”. Thus, models that can classify the character of the entity into “B-^*∗*^/I-^*∗*^” correctly is useful and appreciated more than the models that can accurately classify the character of the entity into “O”. Thus, to verify this ability of the representative models, we complete the experiments in the identification way. The identification F1-scores of all comparison models are shown in Figure 3. As shown in Figure 3, all models obtain improvements in identification than classification, which means the ratio of correctly classifying the true entities is larger than the ratio of correctly classifying the true nonentities. On the publication dataset (the left two pictures), the improvement of RoBERTa-c between identification and classification is the smallest when compared with other representative models. It demonstrates that this model has the stability in identifying the useful TCM named entity, which shows the effectiveness of the word-character integrated self-attention module. The BERT-BiLSTM-CRF model's performance decreases from 96.1 to 75.3 on disease category, which means the ratios of both misclassifying the “O” entities and “B-^*∗*^/I-^*∗*^” entities are relatively high. The same situation about BERT-BiLSTM-CRF also happened on the medical records dataset. On the medical record dataset (the right two pictures), the RoBERTa-c still gains consistent performance. We notice that all models in this experiment obtain relatively large improvements on the medical record dataset than the publication dataset, which means that all models fit less well on the medical records dataset than the publication dataset. However, considering that all models are trained without any samples that come from the medical record dataset, the language-model-based models actually obtain promising performance, especially the model with the word-character integrated self-attention module. We also notice that the performances of all models on treatment law and herb are both higher than other types of entities, especially in medical records. This is mainly because of the normalization of these two types of entities. These two types of entities are usually more standardized terms, while the other three types are more irregular, especially for the clinical manifestation entities.

## 4. Conclusions

In this work, we work with the TCM doctors and experts to collect a publication dataset and a medical record dataset to fill the gap of lacking the comprehensive TCM NER datasets. These datasets contain not only the standard contents that are extracted from the books and articles but also the clinical electronic medical records, which pose the more challenging datasets for TCM NER. We systematically define the 5 types of TCM named entity according to all aspects of TCM diagnosis and treatment, called **CSDTH** classification strategy. The **CSDTH** includes the Clinical manifestation (the pathological information collection), Syndrome (the TCM diagnosis of the course of the disease), Disease (the diagnosis of TCM disease), Treatment law (the decision of treatment principles), and Herb (the concretely used medicines). To handle the variable length of the potential entities, we argue that the character-level representation and tagging might be more suitable for the TCM NER task and propose a word-character integrated self-attention module to generate a new level character representation. The exhaustive experiments demonstrate the effectiveness of the proposed module and the pros and cons of different models.

## Figures and Tables

**Figure 1:** The overall process of generating the new character-level representation.

**Figure 2:** The word semantic and word-character semantic relation integrated character-level representation generation process. The character-level representation is used as the *key* and *value* of the multihead self-attention. The word/phrase-level representation is explored as the *query* of the multihead self-attention.

**Figure 3:** The classification and identification experiments of the representative models on the test set of publications and medical records. All compared models achieve a better performance in the way of identification than classification. It shows that all models misclassify the character that its gold label is “O” into “B-^*∗*^/I-^*∗*^. We notice that the difference of RoBERTa-c between classification and identification is the smallest.

**Table 1:** An example of the TCM clinical records.

Item	Content
Clinical manifestation	Insomnia, dreaminess, palpitation, amnesia, dry stool and once every 2 days, wheezing due to retention of phlegm in throat, palms and soles, dysphoria with feverish sensation in chest, tidal fever, night sweating, red tongue, less tongue coating, small and weak pulse
Syndrome	Heart yin injury, the insufficiency of blood and body fluid, hyperactivity of fire due to yin deficiency
Disease	Insomnia
Treatment law	Nourishing yin and the blood, easing mental anxiety
Herbs	Radix Rehmannia preparata, *Asparagus cochinchinensis*, Radix Scrophulariae, Radix Ginseng, *Poria cocos*, Chinese angelica, Semen Platycladi, Semen ziziphi spinosae, polygala root, the root of red-rooted salvia, the fruit of Chinese magnolia vine

The main content contains 5 terms: clinical manifestation, syndrome, disease, treatment law, and herbs. Other side information, such as a patient's name and age, is omitted.

**Table 2:** The named entity tags used in this work.

Entity type	Clinical manifestation	Syndrome	Disease	Treatment law	Herb	Others
Tags	B-symptom, I-symptom	B-syndrome, I-syndrome	B-disease, I-disease	B-treatment law, I-treatment law	B-herb, I-herb	O

**Table 3:** The statistics of the PubMed dataset.

	Train set	Valid set	Test set
Clinical manifestation	24332	8111	8111
Syndrome	7613	2538	2538
Disease	2808	935	935
Treatment law	11186	3728	3728
Herb	11682	3627	3627
Total	56,628	18,876	18,876

**Table 4:** The number of entities of 5 classes.

Dataset	Number of entities						Number of samples
	Clinical manifestation	Syndrome	Disease	Treatment law	Herb	Total	
Publications	18,150	9,043	1,327	10,698	9,689	48,907	79579
Medical records	75,177	37,053	1,428	9,968	57,836	181,462	14801

**Table 5:** The performances of different models in the test set of publications and the entire medical records.

%	Publications (test)			Medical records		
	P	R	F1	P	R	F1
BiLSTM-CRF	60.8	30.6	40.7	61.4	48.3	54.1
BERT-CRF	58.7	54.2	56.4	54.7	60.5	57.4
BERT-BiLSTM	93	91.6	90.3	85.5	88.1	86.8
BERT-BiLSTM-CRF	75.4	73.1	74.2	69	75.2	71.9
RoBERTa-BiLSTM	88.8	92.6	90.7	86.3	90.1	88.2
RoBERTa-c	92.6	96.7	94.6	90.4	92.3	91.3

**Table 6:** The ablation study for all comparison models.

F1-score (%)	Clinical manifestation		Syndrome		Disease		Treatment law		Herb		Total	
	Publications (test)	Medical records	Publications (test)	Medical records	Publications (test)	Medical records	Publications (test)	Medical records	Publications (test)	Medical records	Publications (test)	Medical records
BERT-BiLSTM-CRF	75.1	55.7	76.9	63.2	73.6	59.6	78.9	68.1	76	79.2	74.2	71.9
BERT-BiLSTM-CRF-c	79.6	60.3	80.3	70.4	78.2	63.4	81.5	73.3	81.2	82.6	79.5	76.4
BERT	94	76.2	91.2	73.7	86.7	76.6	94.3	87.1	93.4	93.4	89.3	86.4
BERT-c	95.2	79.4	94.3	76.8	88.4	76.6	96.5	90.2	94.4	95.2	90.8	88.6
BERT-LSTM	89.3	74.3	90.3	71.2	88	74.2	90.6	85.4	88.4	92.5	86.2	85.1
BERT-LSTM-c	91.3	76.2	92.3	73.5	89.1	74.2	92.7	87.3	90.1	93.6	88.6	87.3
BERT-BiLSTM	94	77.3	93.5	78.4	93	75.7	94.1	83.2	93.3	92.9	90.3	86.8
BERT-BiLSTM-c	94.9	78.3	94.1	79.6	93.5	75.7	94.9	84	94.3	93.9	92.3	87.1
RoBERTa	96.5	81.5	94.2	80.3	96.9	80.7	96.2	**95.3**	96.3	95	92.9	89.5
RoBERTa-c	**98.3**	**83.9**	**97.1**	**85.5**	**98.6**	**81.8**	**98.8**	94.2	**98.7**	**97.9**	**94.6**	**91.3**
RoBERTa-LSTM	94.2	78.1	92.8	77.5	94.5	78.6	94.2	88.3	93.5	94.5	90.3	87.8
RoBERTa-LSTM-c	95.1	79.5	94.2	79.6	95.7	78.6	96	89.6	94.8	96.1	91.7	89.6
RoBERTa-BiLSTM	94.5	78.7	95.1	79.3	95.4	79.6	94.7	88.9	94.3	94.7	90.7	88.2
RoBERTa-BiLSTM-c	94.9	79.1	95.9	80.4	96.1	79.6	95.8	89.7	95.3	95.2	92.3	88.5

The model with “-c” suffix means this model has the word-character integrated self-attention module.

## Data Availability

The datasets used to support the findings of this study are available from the corresponding author upon request.

## References

[1] Fang S., Dong L., Liu L. (2020). HERB: a high-throughput experiment- and reference-guided database of traditional Chinese medicine. *Nucleic Acids Research*.

[2] Yoo M., Shin J., Kim H. (2019). Exploring the molecular mechanisms of traditional Chinese medicine components using gene expression signatures and connectivity map. *Computer Methods and Programs in Biomedicine*.

[3] Xu H.-Y., Zhang Y.-Q., Liu Z.-M. (2019). ETCM: an encyclopaedia of traditional Chinese medicine. *Nucleic Acids Research*.

[4] Xu Q., Tang W., Teng F. (2019). Intelligent syndrome differentiation of traditional Chinese medicine by ANN: a case study of chronic obstructive pulmonary disease. *IEEE Access*.

[5] Na D., Xu C., Caiquan X. A method of collecting four character medicine effect phrases in TCM patents based on semi-supervised learning.

[6] Helfenstein A., Tammela P. (2017). Analyzing user-generated online content for drug discovery: development and use of MedCrawler. *Bioinformatics*.

[7] Liu G.-P., Yan J.-J., Wang Y.-Q. (2014). Deep learning based syndrome diagnosis of chronic gastritis. *Computational and mathematical methods in medicine*.

[8] Liu Z., Zheng Z., Guo X. (2019). AttentiveHerb: a novel method for traditional medicine prescription generation. *IEEE Access*.

[9] Hu Y., Wen G., Liao H. (2019). Automatic construction of Chinese herbal prescriptions from tongue images using CNNs and auxiliary latent therapy topics. *IEEE transactions on cybernetics*.

[10] Tago K., Wang H., Jin Q. Classification of TCM pulse diagnoses based on pulse and periodic features from personal health data.

[11] Weng H., Liu Z., Maxwell A. Multi-label symptom analysis and modeling of TCM diagnosis of hypertension.

[12] Peng Y., Tang C., Chen G. Multi-label learning by exploiting label correlations for TCM diagnosing Parkinson’s disease.

[13] Zhang T., Wang Y., Wang X. (2020). Constructing fine-grained entity recognition corpora based on clinical records of traditional Chinese medicine. *BMC Medical Informatics and Decision Making*.

[14] Zhang D., Xia C., Xu C. (2020). Improving distantly-supervised named entity recognition for traditional Chinese medicine text via a novel back-labeling approach. *IEEE Access*.

[15] Wang Y., Sun Y., Ma Z., Gao L., Xu Y. (2020). Named entity recognition in Chinese medical literature using pretraining models. *Scientific Programming*.

[16] Song B., Bao Z., Wang Y. Incorporating lexicon for named entity recognition of traditional Chinese medicine books.

[17] Qu Q., Kan H., Wu Y., Gao Y. Named entity recognition of TCM text based on Bert model.

[18] Lin F., Xie D. Research on named entity recognition of traditional Chinese medicine electronic medical records.

[19] Gong L., Zhang Z., Chen S. (2020). Clinical named entity recognition from Chinese electronic medical records based on deep learning pretraining. *Journal of Healthcare Engineering*.

[20] Yin M., Mou C., Xiong K. (2019). Chinese clinical named entity recognition with radical-level feature and self-attention mechanism. *Journal of Biomedical Informatics*.

[21] Jin Z., Zhang Y., Kuang H. Named entity recognition in traditional Chinese medicine clinical cases combining BiLSTM-CRF with knowledge graph.

[22] Liu L., Wu X., Liu H. (2020). A semi-supervised approach for extracting TCM clinical terms based on feature words. *BMC Medical Informatics and Decision Making*.

